# Association between Oxidative Burden and Restenosis: A Case-Control Study

**DOI:** 10.1155/2022/3577761

**Published:** 2022-06-28

**Authors:** Shiva Ganjali, Atena Mansouri, Mitra Abbasifard, Seyed Adel Moallem, Zahra Tayarani-Najaran, Amirhossein Sahebkar

**Affiliations:** ^1^Department of Medical Biotechnology and Nanotechnology, Mashhad University of Medical Sciences, Mashhad, Iran; ^2^Biotechnology Research Center, Pharmaceutical Technology Institute, Mashhad University of Medical Sciences, Mashhad, Iran; ^3^Cellular & Molecular Research Center, Birjand University of Medical Sciences, Birjand, Iran; ^4^Immunology of Infectious Diseases Research Center, Research Institute of Basic Medical Sciences, Rafsanjan University of Medical Sciences, Rafsanjan, Iran; ^5^Department of Internal Medicine, Ali-Ibn Abi-Talib Hospital, School of Medicine, Rafsanjan University of Medical Sciences, Rafsanjan, Iran; ^6^Department of Pharmacology and Toxicology, College of Pharmacy, Al-Zahraa University for Women, Karbala, Iraq; ^7^Department of Pharmacodynamics and Toxicology, School of Pharmacy, Mashhad University of Medical Sciences, Mashhad, Iran; ^8^Targeted Drug Delivery Research Center, Pharmaceutical Technology Institute, Mashhad University of Medical Sciences, Mashhad, Iran; ^9^Medical Toxicology Research Center, Mashhad University of Medical Sciences, Mashhad, Iran; ^10^Applied Biomedical Research Center, Mashhad University of Medical Sciences, Mashhad, Iran; ^11^Department of Biotechnology, School of Pharmacy, Mashhad University of Medical Sciences, Mashhad, Iran

## Abstract

**Background:**

In-stent restenosis (ISR) is an important clinical complication that occurs following stent implantation. The application of drug-eluting stents (DES) and even consumption of drugs such as antiplatelet agents and statins are not completely effective in reducing ISR risk. Since the number of these patients continues to rise, it is pivotal to detect patients who are at a higher risk of ISR. In addition, identification of biochemical markers of ISR could give the right perspective on choosing the proper strategy to treat these patients. Several pathophysiological pathways including oxidative stress (OS) are implicated in the progression of ISR. Hence, this study aimed to evaluate the association between oxidative/anti-oxidative markers and ISR.

**Methods:**

This was a case-control study which comprised 21 ISR, 26 NISR (non-ISR), and 20 healthy subjects. The serum levels of OS markers including malondialdehyde (MDA), thiol groups (GSH), total antioxidant capacity (TAC), and the activity of serum antioxidant enzymes such as glutathione peroxidase (GPx) and superoxide dismutase (SOD) were assessed by colorimetric methods. The overall oxidative burden was assessed using a pro-oxidant-antioxidant balance (PAB) assay.

**Results:**

MDA levels were considerably higher in the ISR group when compared to healthy subjects (*P* = 0.004). PAB also indicated significantly higher values in both ISR (*P* < 0.001) and NISR (*P* < 0.001) groups related to healthy subjects. No significant differences were observed between the studied groups regarding thiol levels, antioxidant enzyme activities, and TAC. Multinomial logistic regression analysis showed that elevated serum levels of MDA (OR: 1.028, 95% CI: 1.008-1.048; *P* = 0.006) and PAB (OR: 1.076, 95% CI: 1.017-1.139; *P* = 0.011) were significantly associated with higher ISR risk; however, increased values of TAC (OR: 0.990, 95% CI: 0.982-0.999; *P* = 0.030) were significantly associated with decreased ISR risk, while after adjustment for confounders, only SOD activity (OR: 0.0, 95% CI: 0.0-0.0; *P* < 0.001) and PAB value (OR: 1.866, 95% CI: 1.856-1.900; *P* < 0.001) showed association with ISR risk.

**Conclusion:**

According to the present findings, some oxidative and antioxidative markers like PAB and SOD activity showed the potential in the prediction of ISR risk.

## 1. Introduction

Atherosclerotic cardiovascular disease (ASCVD) is one of the main causes of mortality worldwide [1]. Percutaneous coronary intervention (PCI) with stent implantation is one of the most effective approaches to restore coronary blood flow in atherosclerosis, especially in high-risk patients for whom coronary artery bypass surgery may be considered threatening. However, in-stent restenosis (ISR) is a principal clinical drawback occurring in these patients [2, 3].

Despite many advances in this field like the use of drug-eluting stents (DES) and antiplatelet agents that reduce neointimal hyperplasia to some extent, ISR still remains a major clinical problem occurring in patients who undergo stent implantation [4, 5]. Since the number of these patients continues to rise, it is pivotal to identify patients who are at a higher risk of ISR. In fact, identification of biochemical markers of ISR could give the right perspective on choosing the proper strategy to treat these patients in order to lessen the need for reintervention, improve patient outcomes, and reduce healthcare costs.

Several pathophysiological pathways including alterations of plasma lipids and lipoproteins, endothelial dysfunction, chronic vascular inflammation, elevated oxidative stress (OS), and diminished redox processes are involved in the progression of ISR [4, 6, 7]. Tissue injury followed by stent implantation may lead to increased production of reactive oxygen species (ROS) that contribute to the initial proliferation, migration, and apoptosis of vascular smooth muscle cells as part of the restenosis progression [8–10]. On the other hand, the capacity of intrinsic antioxidant defense system as vascular repair responses in tissue damage [9] has been suggested to be diminished in restenosis. In this regard, the association between reduced glutathione peroxidase (GPx) activity, as well as increased lipid peroxidation with ISR risk, has been illustrated previously [4, 11].

Therefore, this study aimed to evaluate the association of oxidative/antioxidative markers with ISR, in order to find a sensitive and reliable potential marker for accurate and timely diagnosis of patients who are at increased risk of ISR.

## 2. Material and Methods

### 2.1. Study Population

This was a case-control study performed between December 2014 and April 2017, and based on nonprobability (purposive) sampling, we enrolled 47 unrelated Iranian patients (18-75 years old) with a history of coronary angioplasty with stent implantation at least 1 month earlier who were eventually returned due to the chest pain or equivalent symptoms. According to the angiographic results, patients who had >50% and <50% stenosis within the stent were placed into the in-stent restenosis (ISR; *N* = 21) and non-ISR (NISR; *N* = 26) groups, respectively. Patients with primary PCI, positive troponin, and restenosis in the first month after angioplasty due to thrombosis, autoimmune disorder, active cancer, thrombophilia, or chronic kidney disease were excluded. Furthermore, 20 healthy controls were considered as a validation group. Demographic data including sex, age, smoking history, drug history, past history of diabetes mellitus (DM), hypertension (HTN), dyslipidemia, and duration between coronary stenting and subsequent angiography were collected from medical records. The study protocol was given approval by the Ethics Committee of the Mashhad University of Medical Sciences, and written informed consent was obtained from all participants. Inclusion and exclusion criteria were defined previously [12]. Peripheral femoral or brachial blood was drawn right after entering the catheter; serum samples were separated immediately by centrifugation (20 min, 1000 RCF) and then stored at –80 °C until further investigation. Biochemical analysis including fasting blood glucose (FBG), triglycerides (TG), total cholesterol (TC) and high-density lipoprotein cholesterol (HDL-C) was performed by commercial kits (Pars Azmoon, Iran) according to the previously described method [12]. Low-density lipoprotein cholesterol (LDL-C) was calculated using the Friedewald formula.

### 2.2. Assessment of Oxidative Stress and Antioxidant Markers

The serum levels of OS markers including malondialdehyde (MDA) (nmol/mL), thiol groups (GSH) (uM), and total antioxidant capacity (TAC) and the activity of serum antioxidant enzymes such as glutathione peroxidase (GPx) (mU/mL) and superoxide dismutase (SOD) (U) were assessed by colorimetric methods using commercial kits (Kiazist, Iran) according to the manufacturer's protocol as describe in our previous article [13]. Pro-oxidant-antioxidant balance (HK unit) was also measured using a pro-oxidant-antioxidant balance (PAB) assay according to the previously described method [14].

### 2.3. Total Antioxidant Capacity (TAC) Assay

In addition, total antioxidant capacity (TAC) was measured by CUPric Reducing Anti-oxidant Capacity kit (CUPRAC assay kit) (Kiazist, Iran) in accordance with the manufacturer's protocol. In this assay, in the presence of antioxidants, cupric (Cu^2+^) is reduced to cuprous (Cu^+^), and the color which is produced in the presence of chromogen is recorded at 450 nm. TAC was calculated based on a standard curve constructed by Trolox standard available in the kit and was reported as nmol of Trolox equivalent/mL.

### 2.4. Statistical Analysis

SPSS software, version 11.5 (Chicago, IL, USA) was used for statistical analysis. Normal distributed variables which are tested using the Kolmogorov–Smirnov test are presented as mean ± standard error (SE), and one-way analysis of variance (ANOVA) and the Tukey multiple comparison post-test or independent sample *t*-test were used to distinguish changes in variables between the groups. In addition, Chi squared analysis and Fisher's exact test were applied for comparison of qualitative variables between the groups. Binary logistic regression was used to estimate the association between OS markers with ISR (ref: NISR) after adjustment for age, sex, low-density lipoprotein cholesterol (LDL-C), high-density lipoprotein cholesterol (HDL-C) and fasting blood glucose (FBG) levels, Stent type, and use of statins. Moreover, multinomial logistic regression was used to estimate the association between OS markers with ISR (ref: healthy) and NISR (ref: healthy) after adjustment for age, LDL-C, HDL-C, and FBG levels. *P* < 0.05 were considered statistically significant.

## 3. Results

### 3.1. Baseline Characteristics of Subjects

67 participants were enrolled. 20, 26, and 21 were classified into healthy, NISR, and ISR groups, respectively. Groups were not different in terms of gender, although the healthy group included younger individuals in comparison with ISR (*P* < 0.001) and NISR (*P* < 0.001) groups. Significantly great levels of FBG were observed in both ISR (*P* = 0.006) and NISR (*P* = 0.043) groups relative to healthy subjects. Triglyceride (TG) concentrations also showed higher levels in ISR group when compared to NISR (*P* = 0.048) and healthy (*P* = 0.036) groups. The levels of TC (*P* = 0.015), LDL-C (*P* = 0.035), and HDL-C (*P* < 0.001) were significantly higher in healthy individuals in comparison with NISR group. In addition, a higher level of HDL-C was also found in the healthy group when compared to ISR group (*P* = 0.005) (Table 1).

Moreover, the percentage of patients with DES was significantly higher in the NISR group related to the ISR group (Table 2). Totally, most (71.9%) of the patients (the sum of both ISR and NISR) underwent DES implantation, although about half of them (44.7%) had experienced ISR complications.

### 3.2. Oxidative Stress Marker Comparison between the Groups

Serum MDA levels were significantly higher in ISR group in comparison with healthy subjects (*P* = 0.004) (Figure 1). PAB also showed greater levels in both ISR (*P* < 0.001) and NISR (*P* < 0.001) groups when compared to healthy subjects (Figure 2). However, no significant differences in the activities of the antioxidant enzymes GPx and SOD (Figures 3(a) and 3(b), respectively), in thiol levels (Figure 3(c)), and in TAC (Figure 3(d)) were found between the studied groups.

The results of binary logistic regression also failed to show any association between OS markers as well as antioxidant enzyme activities with ISR (reference group: NISR), even after adjustment for age, sex, LDL-C, HDL-C and FBG levels, stent type, and use of statins as confounder factors (Table 3). While multinomial logistic regression showed that elevated levels of MDA (OR: 1.028, 95% CI: 1.008-1.048; *P* = 0.006) and PAB (OR: 1.076, 95% CI: 1.017-1.139; *P* = 0.011) were significantly associated with higher ISR risk (reference group: healthy), increased values of TAC (OR: 0.990, 95% CI: 0.982-0.999; *P* = 0.030) were significantly associated with decreased ISR risk. After adjustment for age, LDL-C, HDL-C, and FBG levels, only elevated PAB and lower SOD activity showed an association with increased ISR risk (Table 4).

High levels of MDA (OR: 1.023, 95% CI: 1.004-1.043; *P* = 0.019) and PAB (OR: 1.094, 95% CI: 1.030-1.162; *P* = 0.004) were also significantly related to the NISR risk. After adjustment for age, LDL-C, HDL-C, and FBG levels, only elevated PAB and lower SOD activity showed an association with increased NISR risk (Table 4).

## 4. Discussion

It is widely accepted that OS, as an imbalance between pro-oxidants and antioxidants [15], is a major factor involved in the vascular injury that leads to the initiation and progression of ASCVD [15]. In this study, for the first time, several oxidative and antioxidative markers were evaluated simultaneously in Iranian patients who underwent stent implantation. The results indicated some changes in OS markers in patients with ISR. Considerably higher levels of MDA were found in the ISR group compared to the healthy subjects. PAB also illustrated significantly higher values in both ISR and NISR groups compared with the healthy individuals. However, no significant differences were observed between the studied groups regarding other OS markers including thiol levels, antioxidant enzyme activities, and TAC. Previously, an increase in markers of OS has been observed after coronary stent implantation, suggesting OS as a trigger of a complex chain of events leading to restenosis [16, 17]. Limitations of the evaluation of MDA, which showed a higher levels in ISR patients compared to the healthy group, have been discussed; however, the test is very simple, rapid, inexpensive, and relatively reliable [18]. Several studies have shown that the plasma levels of TBARS are significantly elevated in patients with ischemic heart disease [19, 20], and it has been suggested that measurement of this parameter may be clinically useful. In fact, significantly higher levels of MDA were observed in patients with angiographically diagnosed coronary artery disease (CAD) relative to the healthy subjects [21]. Moreover, TBARS levels are significantly higher in patients with restenosis after coronary balloon angioplasty [22]. MDA is one of the most commonly used biomarkers for lipid peroxidation, which is associated with atherosclerosis progression [23]. Increase in serum levels of MDA suggests lipid peroxidation of biological membranes and/or lipoproteins in ISR patients. This hypothesis is supported by previous studies, which have shown the presence of elevated levels of antioxidized LDL antibodies in patients at a high risk for restenosis [24].

The activity of the enzyme Gpx, which protects against lipid peroxidation through reduction of free hydrogen peroxide and lipid hydroperoxides [25], showed no significant difference between the studied groups. In contrast, other authors have demonstrated decreased activity of Gpx in ISR groups in comparison with normal controls [4], as well as in human atherosclerotic tissue [26]. Even the activity of SOD, another endogenous enzymatic free radical scavenger which can efficiently detoxify generated ROS [27], showed no statistically significant differences between our studied groups. Our results on SOD are compliant with previous studies in which no differences between ISR, NISR, and normal controls have been demonstrated [4]. The levels of total thiol content and TAC indicated decreased values in ISR and NISR groups compared with the healthy subjects, but the differences were not statistically significant. Other authors have shown lower thiols [21] and lower TAC levels in CAD patients relative to healthy individuals [28]. The discrepancies might be due to the larger sample size of the referred study relative to the current one. On the other hand, the results of PAB assay, which determines the pro-oxidant burden and antioxidant capacity in a single assay [15], revealed an increase in both ISR and NISR groups, when compared to healthy individuals. Increased values of PAB were observed in patients with CAD compared with healthy subjects and a correlation with the severity of angiographic findings was found [15]. Although antioxidant enzyme activities and TAC had not shown any significant alteration between the groups of this study, elevated value of PAB in ISR and NISR patients might be due to the increased pro-oxidant burden in these patients. Moreover, the results of multinomial logistic regression showed that elevated levels of MDA and PAB and decreased levels of TAC were significantly associated with increased risk of ISR. After adjustment for age, LDL-C, HDL-C, and FBG levels, only elevated PAB and lower SOD activity showed a significant association with increased ISR risk. As reported previously, OS levels represented a strong and independent prognostic predictor of cardiovascular events in patients with CAD [29, 30].

The pleiotropic actions of statins have been previously reported [31–40]. Among these pleiotropic activities are antioxidant effects [41]. Through reduction of superoxide anion formation, increasing eNOS activity, and direct antioxidant activity, statins could decrease OS burden [42–46]. Hence, pre-PCI statin therapy could reduce the major adverse cardiac events including death, MI, and target vessel revascularization [47]. In this study, most of the patients in both ISR and NISR group were on statin medication, which might be the reason for increased antioxidant status in patients as high as healthy subjects. Nevertheless, when the use of statins was considered a confounding variable, the results of multinomial logistic regression just showed a significant association between higher MDA levels and higher ISR risk (OR: 1.049, 95% CI: 1.00-1.099; *P* = 0.048) as well as between higher PAB values and higher NISR risk (OR: 1.587, 95% CI: 1.551-1.623; *P* < 0.001) (data are not shown). In addition, the use of DES in patients who undergo angioplasty therapy could reduce the ISR risk by 30-40% [48, 49]. In the United States, the estimated ISR rate is about 10% [50]. In this study, the number of patients who underwent DES implantation was about 71.9%, though about half of them had experienced ISR complications. Nevertheless, when stent type was considered a confounding parameter, the results of binary logistic regression failed to show any association between OS markers as well as antioxidant enzyme activities with ISR. This might be due to the other characteristics of stents like the size and brand of DESs. This information was not available for our studied patients, and this was a limitation of this study. Furthermore, the small sample size of this study along with the lack of sufficient data regarding other confounders like restenosis in more than one stent, *de novo* stenosis in other vessels, and vessel caliber were other limitations of the current study. In addition, the current findings are confined to the Iranian population and further supportive evidence from other ethnic groups is warranted.

In conclusion, according to our findings, oxidative and antioxidative markers could not distinct ISR from NISR; however, variables like PAB and SOD activity showed a potential for the prediction of both ISR and NISR risk. Therapeutic strategies addressing ROS production and antioxidant systems may prevent OS and complications like ISR in patients who undergo stent implantation. To verify this hypothesis, interventional and prospective studies with larger sample sizes are needed.

## Figures and Tables

**Figure 1:** Comparison of the MDA levels between the studied groups. Data are expressed as mean ± SE. ∗∗*P* < 0.01. MDA: malondialdehyde; ISR: in-stent restenosis; NISR: non-in-stent-restenosis.

**Figure 2:** Comparison of the PAB between the studied groups. Data are expressed as mean ± SE. ∗∗∗*P* < 0.001. PAB: pro-oxidant-antioxidant balance.

**Figure 3:** Comparison of the (a) GPx activity; (b) SOD activity; (c) total thiol content of serum; (d) TAC of serum between the studied groups. Data are expressed as mean ± SE. GPX: glutathione peroxidase; SOD: superoxide dismutase; TAC: total antioxidant capacity.

**Table 1:** Baseline characteristics of subjects.

	Healthy (*n* = 20)	NISR (*n* = 26)	ISR (*n* = 21)	*P* value
Sex (%)				
Male	8 (40%)	13 (50%)	11 (52.4%)	0.700
Female	12 (60%)	13 (50%)	10 (47.6%)	
Age (y)	34.50 ± 1.70^a,b^	60.38 ± 2.14	59.48 ± 2.60	0.000∗
FBG (mg/dL)	90.60 ± 1.24^a,b^	138.90 ± 15.72	155.62 ± 17.00	0.006∗
TC (mg/dL)	155.50 ± 5.10^b^	124.40 ± 8.74	145.62 ± 7.90	0.016∗
LDL-C (mg/dL)	93.40 ± 5.72^b^	70.84 ± 6.40	81.70 ± 6.70	0.045∗
TG (mg/dL)	91.80 ± 4.54^a^	97.31 ± 11.80^a^	144.80 ± 21.20	0.022∗
HDL-C (mg/dL)	46.90 ± 2.40^a,b^	34.11 ± 2.20	36.60 ± 1.64	0.000∗

Data are shown as mean ± SE or number (percentage). ^a^Significant in comparison with ISR group. ^b^Significant in comparison with NISR group. IRS: in-stent restenosis; NISR: non-in-stent restenosis; FBG: fasting blood glucose; TC: total cholesterol; LDL-C: low-density lipoprotein cholesterol; TG: triglycerides; HDL-C: high-density lipoprotein cholesterol.

**Table 2:** Clinical characteristics of ISR and NISR groups.

Variables	ISR (*n* = 21)	NISR (*n* = 26)	*P* value
Dyslipidemia %	71.4	46.2	0.081
Diabetics %	61.9	46.2	0.282
Hypertension %	71.4	65.4	0.659
Stent type %			
Bare	50.0	11.1	0.015^∗^
Drug	50.0	88.9	
Stent number %			
1	66.7	65.4	0.927
>1	33.3	34.6	
De novo stenosis in other vessels %	57.1	60.9	0.802
Duration of stent implantation (month)	32.8 ± 5.9	22.4 ± 5.4	0.200
Ejection fraction (%)	46.2 ± 2.9	45.2 ± 2.5	0.806
hs-CRP (mg/L)	3.90 ± 0.8	4.62 ± 0.8	0.509
Drugs consumption %			
Statin	100.0	88.0	0.239
Aspirin	90.5	84.0	0.257
Clopidogrel	68.4	92.0	0.095
NSAID	15.0	4.0	0.197
*β* blocker	5.9	12.5	0.555
ARB	58.8	50.0	
ACE inhibitor	29.4	12.5	
CCB	5.9	18.8	
Insulin	19.0	19.2	0.324
Oral diabetic drugs	38.1	19.2	

Data are expressed as mean ± SE or percentage; ^∗^statistically significant (*P* < 0.05). ISR: in-stent restenosis; NIRS: non-in-stent restenosis; hs-CRP: high-sensitivity C-reactive protein; ARB: angiotensin receptor blockers; ACE: angiotensin converting enzyme; CCB: channel calcium blocker; NSAID: nonsteroidal anti-inflammatory drugs.

**Table 3:** Binary logistic regression for oxidative stress markers in relation to ISR (Ref: NISR).

Variables	ISR			
	Unadjusted		Adjusted^#^	
	OR (95% CI)	*P* value	OR (95% CI)	*P* value
GPX activity (mU/mL)	1.003 (0.915-1.100)	0.947	1.249 (0.870-1.794)	0.228
MDA concentration (nmol/mL)	1.004 (0.995-1.013)	0.347	0.986 (0.958-1.015)	0.341
SOD activity (U)∗	1.077 (0.709-1.636)	0.727	0.995 (0.367-2.694)	0.992
Thiol concentration (uM)	0.998 (0.993-1.003)	0.436	0.994 (0.984-1.005)	0.268
TAC (nmol of Trolox equivalent/mL)	0.997 (0.990-1.004)	0.432	0.991 (0.976-1.006)	0.242
PAB (HK unit∗∗)	0.984 (0.963-1.006)	0.161	0.996 (0.963-1.030)	0.823

^#^Adjusted for age, sex, LDL-C, HDL-C, and FBG levels, stent type, and use of statins. LDL-C: low-density lipoprotein cholesterol; HDL-C: high-density lipoprotein cholesterol; FBG: fasting blood glucose; ISR: in-stent restenosis; NISR: non-in-stent-restenosis; GPX: glutathione peroxidase; MDA: malondialdehyde; SOD: superoxide dismutase; TAC: total antioxidant capacity; PAB: pro-oxidant-antioxidant balance; OR: odds ratio; CI: confidence interval.

**Table 4:** Multinomial logistic regression for oxidative stress markers in relation to ISR and NISR (ref: healthy).

Variables	NISR				ISR			
	Unadjusted		Adjusted^#^		Unadjusted		Adjusted^#^	
	OR (95% CI)	*P* value	OR (95% CI)	*P* value	OR (95% CI)	*P* value	OR (95% CI)	*P* value
GPX activity (mU/mL)	1.017 (0.909-1.138)	0.771	0.820 (0.455-1.476)	0.507	1.021 (0.910-1.146)	0.722	0.841 (0.467-1.514)	0.564
MDA concentration (nmol/mL)	1.023 (1.004-1.043)	0.019∗	1.026 (0.966-1.089)	0.409	1.028 (1.008-1.048)	0.006∗	1.031 (0.970-1.095)	0.325
SOD activity (U)∗	1.030 (0.602-1.762)	0.915	0.0 (0.0)	0.000∗	1.144 (0.692-1.893)	0.599	0.0 (0.0)	0.000∗
Thiol concentration (uM)	0.999 (0.994-1.004)	0.748	0.988 (0.970-1.006)	0.201	0.995 (0.988-1.003)	0.197	0.985 (0.966-1.003)	0.108
TAC (nmol of Trolox equivalent/mL)	0.994 (0.987-1.002)	0.153	0.987 (0.967-1.008)	0.140	0.990 (0.982-0.999)	0.030∗	0.984 (0.964-1.005)	0.227
PAB (HK unit∗∗)	1.094 (1.030-1.162)	0.004∗	1.891 (1.847-1.935)	0.000∗	1.076 (1.017-1.139)	0.011∗	1.866 (1.856-1.900)	0.000∗

^#^Adjusted for age, LDL-C, HDL-C, and FBG levels. LDL-C: low-density lipoprotein cholesterol; HDL-C: high-density lipoprotein cholesterol; FBG: fasting blood glucose; ISR: in-stent restenosis; NISR: non-in-stent-restenosis; GPX: glutathione peroxidase; MDA: malondialdehyde; SOD: superoxide dismutase; TAC: total antioxidant capacity; PAB: pro-oxidant-antioxidant balance; OR: odds ratio; CI: confidence interval.

## Data Availability

The data are available upon request.

## Abbreviations

ACE: Angiotensin converting enzyme
ANOVA: One-way analysis of variance
ARB: Angiotensin receptor blockers
CCB: Channel calcium blocker
CI: Confidence interval
CU+: Cuprous
Cu2+: Cupric
CVD: Cardiovascular disease
DES: Drug eluting stents
DM: Diabetes mellitus
FBG: Fasting blood glucose
HDL-C: High-density lipoprotein cholesterol
HK unit: Hamidi-Koliakos unit
HTN: Hypertension
hs-CRP: High-sensitivity C-reactive protein
GSH: Glutathione
GPx: Glutathione peroxidase
ISR: In-stent restenosis
LDL-C: Low-density lipoprotein cholesterol
MDA: Malondialdehyde
mg/dL: Milligrams per deciliter
nmol/mL: Nanomole per milliliter
NIRS: Non-in-stent restenosis
NSAID: Nonsteroidal anti-inflammatory drugs
OR: Odds ratio
OS: Oxidative stress
PAB: Pro-oxidant-antioxidant balance
PCI: Percutaneous coronary intervention
ROS: Reactive oxygen species
SE: Standard error
SOD: Superoxide dismutase
TAC: Total antioxidant capacity
TC: Total cholesterol
TG: Triglycerides
Y: Year.
